The article "Improved Fire Retardancy of Cellulose Fibres via Deposition of Nitrogen-Modified Biopolyphenols" was published in 2022. Journal: Molecules.

# Improved Fire Retardancy of Cellulose Fibres via Deposition of Nitrogen-Modified Biopolyphenols

**DOI:** 10.3390/molecules27123741

**Published:** 2022-06-10

**Authors:** Tiina Pöhler, Petri Widsten, Tuula Hakkarainen

**Affiliations:** VTT Technical Research Centre of Finland Ltd., P.O. Box 1000 Espoo, Finland; petri.widsten@vtt.fi (P.W.); tuula.hakkarainen@vtt.fi (T.H.)

**Keywords:** cellulose, fire performance, fire retardant, lignin, micro-scale combustion calorimetry, modification, nitrogen, pulp, retention aid, tannin

## Abstract

Driven by concerns over the health and environmental impacts of currently used fire retardants (FRs), recent years have seen strong demand for alternative safer and sustainable bio-based FRs. In this paper, we evaluated the potential of nitrogen-modified biopolyphenols as FRs for cellulosic natural fibres that could be used in low-density cellulose insulations. We describe the preparation and characterisation of nitrogen-modified lignin and tannin containing over 10% nitrogen as well as the treatment of cellulose pulp fibres with combinations of lignin or tannin and adsorption-enhancing retention aids. Combining lignin or tannin with a mixture of commercial bio-based flocculant (cationised tannin) and anionic retention chemical allowed for a nearly fourfold increase in lignin adsorption onto cellulosic pulp. The nitrogen-modified biopolyphenols showed significant improvement in heat release parameters in micro-scale combustion calorimetry (MCC) testing compared with their unmodified counterparts. Moreover, the adsorption of nitrogen-modified lignin or tannin onto cellulose fibres decreased the maximum heat release rate and total heat release compared with cellulose reference by 15–23%. A further positive finding was that the temperature at the peak heat release rate did not change. These results show the potential of nitrogen-modified biopolyphenols to improve fire-retarding properties of cellulosic products.

## 1. Introduction

Fibrous cellulosic thermal insulation materials are mainly produced and used in geographical locations such as Scandinavia, Northern America, and Central Europe, where wood-based raw material (recycled newsprint or wood) is abundant. The wood-based insulations in blown or panel form have a comparatively low carbon footprint [1] and their raw material comes mainly from sustainably managed forests either directly or after product (paper) recycling. As the building and construction sector is a major source of CO_2_ emissions globally [2], special attention will be paid in the future to the carbon footprint of single building materials and this may open up new opportunities for cellulosic insulation materials.

Thermal insulations in buildings require appropriate reaction-to-fire properties. Typically, the fire classification of commercial cellulosic insulation is Euroclass E or equivalent, which is the least demanding fire rating among building materials and restricts their use, for example, in multi-story buildings. The ignition time of cellulosic materials decreases as a function of material density [3], showing a clear need for fire retardants (FRs). However, the heat release rate is naturally, without FRs, smaller compared with low density plastic insulation, like expanded polystyrene (EPS) [4,5]. The heat release rate can be further decreased with various types of FRs.

Recent years have seen a growing demand for safer FRs to replace effective, but harmful halogen-based FRs in the construction sector and other sectors [6]. While relatively safe inorganic and inorganic/organic FRs, such as the intumescent FR combination of ammonium polyphosphate and pentaerythritol, are widely used, especially among polyolefins, it is nowadays increasingly regarded that FR raw materials should not be drawn from resources that are used for fertilisers in food production (e.g., phosphates) or require large molar equivalents of synthetic chemicals for production (e.g., pentaerythritol). In this regard, FRs based on technical lignin [7] and tannin [8] present themselves as a more sustainable alternative. Lignin and tannin are phenolic biopolymers with a relatively high carbon content and a good ability to form carbonaceous char. In the event of fire, FR coatings based on lignin and tannin form a layer of char on the surface of the burning material, helping to isolate it from heat, oxygen, and flammable gases of combustion [9]. These insulation properties are enhanced by chemically introduced nitrogen functionalities, giving rise to nitrogen-based gases such as ammonia and nitrogen oxide that make the coatings more intumescent. For lignin, other fire-inhibiting mechanisms have also been put forward [9]. The aromatic units of lignin and tannin can be modified, e.g., by Mannich reaction [4,10] or Michael addition of amino-based nucleophiles [11] to reactive quinone methide intermediates to add nitrogen as amino or urea groups into their polymeric structures, while carbonyl groups occurring on the lignin phenylpropane side chains or as quinones can react with nitrogen nucleophiles such as urea or amines according to the Schiff base reaction to give imines [12]. Although urea and formaldehyde used in the Mannich reaction to add nitrogen to lignin or tannin are synthetic products, and urea is synthesised from ammonia whose main use is in nitrogen-based fertilisers, the polyphenol still comprises nearly 90% of the nitrogen-modified product. Moreover, formaldehyde is produced from methanol that today can be sourced from biorefineries. There are several other routes available for adding nitrogen to biopolyphenols, e.g., polyurethane synthesis [13,14]. 

The ignition and combustion of wood and other cellulosic materials are mainly based on the pyrolysis (i.e., thermal decomposition) of cellulose and the reactions of pyrolysis products with each other and with gases in the air, mainly oxygen. When the temperature increases, cellulose starts to pyrolyse. The decomposition products either remain inside the material or are released as gases. Gaseous substances react with each other and oxygen, releasing a large amount of heat that further induces pyrolysis and combustion reactions.

Depending on environmental conditions such as temperature, oxygen concentration, moisture, fire retardants, pH, and so on, the pyrolysis of cellulose can proceed mainly along two pathways. The tar forming pathway, taking place at a temperature of approximately 300 °C, is related to the normal burning. In this case, pyrolysis produces a lot of tar, including levoglucosan, which decomposes easily to burning gases under the influence of heat. Thermal decomposition can also take place through a char-forming pathway. In this process, cellulose is first transformed to unstable, active cellulose that further decomposes so that the reaction products are mainly carbon dioxide and water, and a backbone of cellulose containing a lot of carbon [15]. Our hypothesis was that the addition of biopolyphenols and especially N-modified biopolyphenols to cellulosic fibres could add to the char-forming process and lessen the formation of levoglucosan. 

The use of organic polymers as FRs in fibrous cellulose insulation materials is uncommon and not straightforward. For example, lignin or other biopolyphenols in powder form could be mixed with dry or wet cellulose fibres, resulting in weak interaction and bonding between the polymeric particles and fibres. Lignobond [16] is a technique that has been used, e.g., in papermaking to deposit high molecular mass lignin tightly onto wet fibre surfaces before material formation in aqueous media. The precipitation of lignin has been shown to improve the strength and water resistance properties of boards or unbleached paper grades. In Lignobond, lignin powder is first dissolved in base and added into the fibre slurry. After mixing, the pH is adjusted to 4.5 with an acid, which starts the precipitation of lignin into solids and onto fibre surfaces. The addition of a cationic and anionic retention aid system into the slurry further improves the retention of lignin onto fibre surfaces. 

We exploited the Lignobond process to add unmodified and nitrogen-modified biopolyphenols, lignin or tannin, onto bleached softwood kraft fibres to investigate their effect on the fire retarding of the cellulosic fibre network. The nitrogen-modification of lignin and tannin was accomplished via Mannich and other reactions by reacting the alkali-dissolved biopolyphenols with urea and formaldehyde. The nitrogen-modified biopolyphenols decreased the heat release rate and total heat release of the cellulose material without changing the temperature at the peak heat release rate. The effect on ignitability was not investigated during this phase.

## 2. Results and Discussion

### 2.1. Nitrogen-Modification of Lignin and Tannin

Adding nitrogen to polyphenols is known to improve their FR properties. Polyphenols with a high nitrogen content can be synthesised using urea and formaldehyde reagents under alkaline conditions [10], whereby multiple reaction routes that result in the introduction of amino or imino groups are available. Unsubstituted aromatic carbons *ortho* or *para* to a phenolic hydroxyl group are potentially reactive sites in the Mannich reaction of lignin and tannin, whereby the most nucleophilic, electron-rich aromatic carbons attack the electrophilic immonium ion intermediate formed by urea and formaldehyde. Such carbons occur in guaiacyl and *p*-hydroxyphenyl units of lignin and A-rings of procyanidin-type condensed tannin. The Mannich reaction of lignin or tannin with urea and formaldehyde gives methyleneurea-substituted lignin, while any carbonyl groups in lignin may undergo Schiff base reaction with urea, which produce imines [10]. Further potential reaction routes are conjugate (Michael) additions of urea to quinone methide intermediates, formed in lignin under alkaline conditions, or to pre-existing ring-conjugated double bonds or quinones [17] in the lignin polymer. These reaction routes are illustrated in Figure 1.

^31^P NMR spectral analysis (Table 1) shows that the nitrogen-modification reduced the guaiacyl and *p*-hydroxyphenyl units of hardwood (HW) kraft lignin in accordance with the mechanism of Mannich reaction [4,10], the amino groups in the product appearing at ca. 133 pm [18] (Figure 2). The number of Mannich reactive sites is approximately the sum of *ortho*-unsubstituted guaiacyl and *p*-hydroxyphenyl hydroxyls, 0.91 mmol/g, which is only 26% of the total phenolic hydroxyls. In the modified lignin, there are only 0.31 mmol/g of these phenolic hydroxyls left—a reduction of 0.60 mmol/g (66%, or a little less if the increase in lignin molar mass resulting from the nitrogen modification is considered). Theoretically, the molar increase in primary and secondary amino groups should be twice the number of reactive sites consumed (excluding the possibility of crosslinking reactions giving diarylmethyl urea), or 1.20 mmol/g, while the measured amino content was slightly higher at 1.47 mmol/g. It is possible that base-catalysed hydrolysis of alkyl–aryl ether linkages liberated more phenolic hydroxyls and increased the number of Mannich-reactive sites during the reaction. Amino groups of imines or other amino-bearing reaction products may also contribute to the signal intensity near 133 pm.

The nitrogen content of the HW kraft lignin increased from negligible to 10% (Table 1). Given the relatively small number of Mannich reactive sites in the lignin, this figure is too high to assume that all of the nitrogen was introduced by the Mannich reaction, as it would correspond to a methyleneurea substituent (MW 73 g/mol) content of 26% in the modified lignin and place the degree of lignin methyleneurea substitution at 1.0 per lignin unit (assuming 200 g/mol for an average phenylpropane unit). It thus seems that urea-based modifications that do not involve formaldehyde (Schiff base reaction and Michael addition) contributed significantly to the introduction of nitrogen in the lignin polymer.

Spruce tannins are predominantly procyanidin-type condensed tannins [19,20]. After correction for non-tannin components amounting to ca. 40%, the N content (Table 1) of the procyanidin component is ca. 17.7%, corresponding to a methyleneurea substituent content of 46% per procyanidin unit, or a substitution rate of 1.2 methyleneurea groups per procyanidin unit (MW 288 g/mol), assuming that only procyanidin units participated in the Mannich reaction. The main sites of reaction are probably the double-activated electron-rich carbons of the A-ring located *ortho*-*ortho* and *ortho*-*para* to the phenolic hydroxyls. While the three unsubstituted carbons of the B-ring are in the *ortho* or *para* position of a phenolic hydroxyl, they are also deactivated by being *meta* to the other phenolic hydroxyl, rendering them considerably less nucleophilic than the double activated A-ring carbons.

### 2.2. Heat Release Properties of Unmodified and N-Modified Biopolyphenols

The peak heat release rate (PHRR), temperature at PHRR (T_PHRR_), and total heat release (THR) of pure lignin and tannin samples were determined by micro-scale combustion calorimetry (MCC). The char yield was determined gravimetrically.

The MCC test results of pure compounds are presented in Table 2 as PHRR, T_PHRR_, THR, and char yield values, and in Figure 3 as HRR as a function of temperature, comparing unmodified and N-modified samples. The repeatability of the replicate tests was found to be good, as can be seen from the scalar values of Table 2. Therefore, only test 1 of each sample is shown in Figure 3 to represent the heat release behaviour in the MCC tests.

For pure lignin, it was observed that N-modification significantly reduced (33–60%) the PHRR value, but bought the peak to a lower temperature. THR was clearly reduced (23–35%) by N-modification. No consistent trend was seen for char yield; the value either increased or decreased depending on the compound.

For spruce tannin, the benefits of N modification for heat release were consistent: PHRR and THR decreased (by 33 and 30%, respectively) and T_PHRR_ increased significantly. Char yield was slightly reduced, but the difference was minor.

### 2.3. Deposited Amounts of Biopolyphenols on Cellulose Kraft Pulp Fibres

A preliminary retention trial (Table 3) was conducted with unmodified HW kraft lignin to select the most promising retention aids for further tests with nitrogen-modified lignin. The retention of lignin on filtrated pulp fibre pads was very low when only lignin was deposited onto the fibres, improving somewhat with the addition of cationic Tanfloc SG. However, the application of Tanfloc SG together with anionic polyacrylamide (A-PAM) allowed for full retention to be achieved. Based on these results, the combination with the highest determined lignin content (2.5% Tanfloc SG + 0.45% A-PAM) was selected for deposition trials with nitrogen-modified biopolyphenols.

The N-modified biopolyphenols were precipitated to bleached SW kraft pulp that itself contained a negligible amount of lignin. Lignin analysis (Table 4) showed that the highest deposited amount was obtained with N-modified HW kraft lignin, that is, 15.9%, and the smallest amount with N-modified spruce tannin, that is, 10.5%. Chemical modification reduced the deposited amount of HW kraft lignin. The dried pulp fibre pads after the Lignobond precipitation with corresponding filtrates are shown in Figure 4. The brown colour of the filtrates resulted from non-adsorbed biopolyphenols.

SEM images taken from the air-dried pulp fibre pads (Figure 5) show the deposited N-modified lignin and tannin particles on the fibre surfaces and in the fibre network. The particles formed crust-like areas on the fibre surfaces and did not fully cover the fibres. The approximate size of the particles lay between 1 and 20 µm, evaluated from the SEM images.

### 2.4. Heat Release Properties of Modified Biopolyphenols Deposited on Cellulose Pulp Fibres

The MCC test results of mixtures with kraft cellulose fibres and Tanfloc SG 2.5% + 0.45% A-PAM are presented in Table 5 as PHRR, T_PHRR_, THR, and char yield values. The repeatability of the replicate tests was not as good as for pure biopolyphenols, as can be seen from the scalar values in Table 5.

The difference between the bleached SW kraft pulp as such and with the retention aid system Tanfloc SG + A-PAM was relatively small. The material with the retention aid system exhibited ca. 5% higher PHRR and THR values than the material without it. Its T_PHRR_ was a few degrees lower. The char yield for both materials was low, ca. 7%.

The addition of N-modified lignin or tannin significantly improved the PHRR and THR values. The reduction of PHRR was 23% for lignin and 17% for tannin compared with the bleached SW kraft pulp reference. THR reduced 13–19% for lignin and 15% for tannin. T_PHRR_ was of the same order for all specimens studied. The char yield was roughly doubled compared with the reference material. Overall, the addition of N-modified biopolyphenols to cellulose fibres had a favourable effect.

## 3. Materials and Methods

### 3.1. Materials

SW (*Pinus sylvestris*/*Picea abies*) and HW (*Eucalyptus* sp.) kraft lignins were industrial lignins precipitated using carbon dioxide from the black liquor of pulp mills that produce paper-grade kraft pulp. SW CatLignin, from *Pinus sylvestris*/*Picea abies*, was produced at a laboratory scale from industrial black liquor using a patented CatLignin method [21] based on heat treatment of black liquor, followed by conventional precipitation using carbon dioxide and acidic washing. Spruce tannin with a tannin content of ca. 60% was prepared by soda cooking of spruce (*Picea abies*) bark followed by acid precipitation (pH 2.5) of tannin from the spent liquor. Tanfloc SG, mimosa tannin cationised with formaldehyde and ammonium chloride [22], was purchased from Christian Markmann GmbH, Hamburg, Germany.

Bleached kraft softwood pulp was obtained from Metsä Fibre Äänekoski mill. Anionic polyacrylamide (A-PAM) was Kemira’s Superfloc A100HMW and aluminium sulphate 18 hydrate was purchased from Acros.

### 3.2. Methods

#### 3.2.1. Nitrogen-Modification of Biopolyphenols

For nitrogen modification of lignin or tannin with urea and formaldehyde, lignin, or tannin, 10.00 g based on oven-dry weight and 10.00 g of urea were placed in a round-bottomed flask equipped with a reflux condenser and dissolved at 70 °C in NaOH solution prepared by combining 210 g of Milli-Q water and 2.0 g of 50% NaOH solution, corresponding to an NaOH dose of 0.65 equivalents per alkali-consuming functional group (hydroxyl and carboxyl). This was followed by the addition of 10 mmol of formaldehyde per 1 g of lignin or tannin, added as 37% aqueous formalin solution (8.1 g) over 10 min. The mixture was refluxed at 70 °C with mechanical stirring for 10 h, after which the product was allowed to cool and then precipitated by first adding 100 mL of water acidified with HCl to pH 3, and then adding concentrated HCl solution dropwise until the pH was lowered to 2–3. The precipitate was washed twice with HCl solution (pH 3) before being freeze-dried.

#### 3.2.2. Chemical Characterisation of Biopolyphenols

The N content was determined using an organic elemental (CHNS) analyser (Flash 2000 Series, Thermo Fisher Scientific BV, Delft, The Netherlands), as described by Nordlund et al. [23]. The hydroxyl and carboxyl contents of lignin were determined from lignin dissolved in pyridine and deuterated chloroform (1.6/1, *v*/*v*) and phosphitylated with 2-chloro-4,4,5,5-tetramethyl-1,3,2-dioxaphospholane by ^31^P NMR on a Bruker Avance III 500 MHz NMR spectrometer at room temperature [24]). *Endo*-N-Hydroxy-5-norbornene-2,3-dicarboximide was used as the internal standard.

#### 3.2.3. Deposition of Biopolyphenols on Cellulose Fibres

Bleached SW kraft pulp was soaked overnight in Milli-Q water, disintegrated at a concentration of 3%, and then further diluted to 1.3%. Table 6 shows the detailed formulation used for Lignobond precipitation. Nitrogen-modified biopolyphenols were dissolved in 0.5 M NaOH. A-PAM was dissolved in 9 mL of Milli-Q water. Then, 150 mL of cellulose fibre slurry was mixed in a decanter glass. The nitrogen-modified biopolyphenols (20% of dry fibre weight) were added to the slurry and the mixture was stirred for 10 min. The pH of the slurry was adjusted to 4.5 with 1 M HCl, after which first Tanfloc SG powder (2.5% on dry fibre) and then A-PAM solution (0.45% on dry fibre) were added as retention aids. The slurry was further mixed for 20 min and then filtered using a wire cloth (mesh size 90 µm). Finally, the wet pulp pad was dried under ambient conditions.

#### 3.2.4. Determination of Pulp Pad Biopolyphenol Content

The lignin/tannin content of pulps was determined as the sum of acid insoluble (Klason) and acid-soluble polyphenols [25]. Klason lignin is the solid residue left after total dissolution of all carbohydrates by 72% sulfuric acid at 20 °C (68 °F) for 2.0 h, followed by dilution to 3% sulfuric acid and refluxing for 4 h. Acid-soluble lignin is determined by UV spectroscopy (UV spectrophotometer: Perkin Elmer Lambda 900, Waltham, MA, USA) from the acid hydrolysis liquid.

#### 3.2.5. Scanning Electron Microscopy

The dry fibre pad sample was attached with double-sided carbon tape to an aluminium sample stub before sputtering a 5 nm layer of Au/Pd with Leica EM ACE200 sputter coater. Secondary electron images with an Everhart–Thornley detector at 1000 times original magnification were collected with a field-emission scanning electron microscope (FE-SEM Merlin, Carl Zeiss Microscopy, Oberkochen, Germany) using an acceleration voltage of 2 kV and probe current of 60 pA.

#### 3.2.6. Micro-Scale Combustion Calorimetry

Micro-scale combustion calorimetry (MCC) is an experimental method for measuring the heat release rate of a small sample (ca. 1–10 mg) as a function of temperature [26,27]. It reveals how much combustible gases evolve and how much energy is released in the pyrolysis of the specimen tested.

In this work, the peak heat release rate (PHRR), temperature at PHRR (T_PHRR_), and total heat release (THR) of lignin and tannin samples were determined by MCC (Govmark Microscale Combustion Calorimeter Model-MCC-2, New York, NY, USA) in a nitrogen atmosphere at a heating rate of 1.4 K/s. The char yield, defined as a percentage by the weight of solid residue remaining after MCC relative to the initial weight of the test specimen, was determined gravimetrically. Two replicate tests were performed for each material.

The MCC measurements performed are considered as an initial screening of the prototype FR systems, the most promising of which are proposed for further evaluation using larger-scale fire test methods, such as the cone calorimeter [28].

## 4. Conclusions

We investigated the potential of safe and renewable biopolyphenols in the fire retarding of another renewable material, cellulose fibres. Our key ideas were the addition of nitrogen to various technical lignin or tannin to enhance their fire-retarding performance, and the deposition of the modified biopolyphenols onto cellulose fibre surfaces by the Lignobond process with a tannin-based retention system. We showed that the N-modification greatly reduced (up to 60%) the specific heat release parameters of the pure biopolyphenols. The effects of modified biopolyphenols on the fire properties of cellulose fibre networks were of a lesser magnitude, but their positive effect was clear. Thus, the results showed their potential to improve the fire-retarding properties of cellulosic products. The decrease in MCC parameters did not reveal the effect of biopolyphenols on the ignitability of cellulose fibre networks, which should be assessed separately.

## Figures and Tables

**Figure 1:** Nitrogen modification of (**A**) tannin and (**B**) lignin aromatic units by Mannich reaction, lignin carbonyls by Schiff base reaction (**C**), Michael addition to ring-conjugated double bonds in lignin side chain (**D**), and Michael addition to quinone methide intermediates in lignin (**E**). Asterisks indicate reactive sites.

**Figure 2:** ^31^P NMR spectra of HW kraft lignin before (**A**) and after (**B**) reaction with urea and formaldehyde. IS = internal standard.

**Figure 3:** Heat release rate (HRR) in the MCC tests of unmodified and N-modified pure compounds: (**a**) SW kraft lignin, (**b**) SW CatLignin, (**c**) HW kraft lignin, and (**d**) Spruce tannin. The result of test 1 is shown for each compound.

**Figure 4:** Pulp fibre pads (top image) and filtrates (bottom image) after LignoBond deposition of N-modified biopolyphenols: (**a**) SW kraft lignin, (**b**) SW CatLignin, (**c**) HW kraft lignin, and (**d**) Spruce tannin.

**Figure 5:** SEM images of pulp fibre pads showing the deposited N-modified lignin and tannin on cellulose fibre surfaces: (**a**) bleached SW kraft pulp (reference), (**b**) +N-modified SW kraft lignin, (**c**) +N-modified SW CatLignin, (**d**) +N-modified HW kraft lignin, and (**e**) +N-modified spruce tannin.

**Table 1:** Functional group (^31^P NMR) and nitrogen (CHNS analysis) content of lignin ^1^ and tannin.

Lignin/Tannin	Carboxyl, mmol/g	Aliphatic Hydroxyl, mmol/g	Phenolic Hydroxyl by Subtype (Lignins Only), mmol/g			Total Phenolic Hydroxyl, mmol/g	Amino, mmol/g	N, %
			Condensedor syringyl	Guaiacyl	p-OH-phenyl			
HW kraft lignin	0.29 ± 0.00	0.95 ± 0.02	2.62 ± 0.09	0.80 ± 0.02	0.11 ± 0.09	3.53 ± 0.13		0.12 ± 0.00
N-modified HW kraft lignin	0.30 ± 0.09	1.02 ± 0.04	2.77 ± 0.02	0.29 ± 0.01	0.02 ± 0.02	2.58 ± 0.05	1.47 ± 0.21	10.12 ± 0.05
Spruce tannin ^3^	1.13 ± 0.02	2.01 ± 0.06				3.49 ± 0.15		0.57 ± 0.01
N-modified spruce tannin ^2^								10.61 ± 0.02
Tanfloc SG								7.60 ± 0.02

^1^ For data on N-modified and unmodified softwood (SW) kraft and SW CatLignin, see [10]; ^2^ insoluble in NMR solvent—spectrum unable to be recorded; ^3^ tannin content 60%.

**Table 2:** MCC test results of pure compounds.

Sample		PHRR (W/g)	T_PHRR_ (°C)	THR (J/g)	Char Yield (wt-%)
SW kraft lignin	Test 1 Test 2 **Average**	121 124 **123**	419 416 **417**	9440 9860 **9650**	38.7 37.7 **38.2**
N-modified SW kraft lignin ^1^	Test 1 Test 2 **Average**	49/48 49/50 **49/49**	269/395 277/402 **273/399**	6340 6200 **6270**	41.6 40.5 **41.0**
SW CatLignin	Test 1 Test 2 **Average**	79 77 **78**	411 413 **412**	6360 6330 **6340**	48.9 49.5 **49.2**
N-modified SW CatLignin	Test 1 Test 2 **Average**	53 52 **52**	285 288 **287**	4860 4920 **4890**	43.8 44.2 **44.0**
HW kraft lignin	Test 1 Test 2 **Average**	154 151 **153**	405 405 **405**	9230 9580 **9400**	36.3 36.2 **36.3**
N-modified HW kraft lignin	Test 1 Test 2 **Average**	64 64 **64**	366 363 **365**	6420 6330 **6370**	39.8 40.0 **39.9**
Spruce tannin	Test 1 Test 2 **Average**	54 55 **55**	256 254 **255**	7280 7300 **7290**	46.1 45.5 **45.8**
N-modified spruce tannin	Test 1 Test 2 **Average**	37 38 **37**	430 413 **422**	5140 5150 **5140**	44.4 44.2 **44.3**

^1^ The sample exhibited two heat release peaks of similar heights. Therefore, two values are presented for PHRR and T_PHRR_.

**Table 3:** Lignin content and filtration retention of bleached kraft pulp combined with HW kraft lignin and retention aids. Mixtures with >95% retention were analysed in triplicate.

Retention Aids	Klason Lignin, % ^1^	Acid-Soluble Lignin, % ^1^	Total Lignin, % ^1^	Retention, % ^2^
None	6.5	0.3	6.8	85.9
Tanfloc SG 2.5%	9.7	0.9	10.7	91.0
Tanfloc SG 2.5%, A-PAM 0.15%	20.0 ± 0.3	3.1 ± 0.1	23.0 ± 0.2	98.4
Tanfloc SG 2.5%, A-PAM 0.30%	22.0 ± 3.2	2.9 ± 0.0	25.0 ± 3.2	103.0
Tanfloc SG 2.5%, A-PAM 0.45%	22.8 ± 0.8	3.3 ± 0.1	26.1 ± 0.7	99.4

^1^ Lignin values include the contribution from Tanfloc SG, if included; ^2^ 100% retention is the sum of fibres, lignin, and retention aids applied.

**Table 4:** Chemical analysis of samples made with the Tanfloc SG 2.5% and A-PAM 0.45% retention system.

Sample	Klason Lignin, %	Acid-Soluble Lignin, %	Total Lignin, %	N, %
Bleached SW kraft pulp	1.2 ± 0.0	0.0 ± 0.0	1.2	0.00 ± 0.00
+N-modified SW kraft lignin	12.5 ± 1.1	1.1 ± 0.0	13.6	1.15 ± 0.13
+N-modified SW CatLignin	11.5 ± 0.6	0.6 ± 0.0	12.1	1.20 ± 0.22
+N-modified HW kraft lignin	14.5 ± 1.0	1.4 ± 0.1	15.9	0.52 ± 0.01
+N-modified spruce tannin	9.8 ± 1.0	0.7 ± 0.0	10.5	0.57 ± 0.02

**Table 5:** MCC test results of mixtures with kraft cellulose fibres and Tanfloc SG 2.5% + 0.45% A-PAM.

Sample		PHRR (W/g)	T_PHRR_ (°C)	THR (J/g)	Char Yield (wt-%)
Bleached SW kraft pulp	Test 1 Test 2 **Average**	315 351 **333**	380 379 **379**	11,360 11,550 **11,460**	6.5 6.6 **6.6**
Bleached SW kraft pulp + retention aid system Tanfloc SG + A-PAM	Test 1 Test 2 **Average**	361 337 **349**	372 371 **372**	12,240 11,870 **12,050**	6.4 7.5 **6.9**
+N-modified SW kraft lignin	Test 1 Test 2 **Average**	268 249 **258**	380 374 **377**	9520 9120 **9320**	15.4 14.4 **14.9**
+N-modified SW CatLignin	Test 1 Test 2 **Average**	265 253 **259**	380 380 **380**	9610 9910 **9760**	14.8 14.5 **14.6**
+N-modified HW kraft lignin	Test 1 Test 2 **Average**	272 242 **257**	386 375 **381**	10,070 9870 **9970**	14.5 12.9 **13.7**
+N-modified spruce tannin	Test 1 Test 2 **Average**	247 303 **275**	371 382 **376**	9280 10,170 **9730**	17.8 14.5 **16.2**

**Table 6:** Formulation in Lignobond precipitation.

	Dry Weight or Volume	% of Pulp Amount
Bleached SW kraft pulp	1.95 g	100
N-modified biopolyphenol	0.40 g	20
0.5 M NaOH	5 mL	
Tanfloc SG	50 mg	2.5
A-PAM	9 mg	0.45

## Data Availability

Not applicable.
